The article "Plasma Methylated RNF180 for Noninvasive Diagnosis of Gastric Cancer" was published in 2022. Journal: Biomed Res Int.

# Plasma Methylated RNF180 for Noninvasive Diagnosis of Gastric Cancer

**DOI:** 10.1155/2022/6548945

**Published:** 2022-10-05

**Authors:** Luyao Zhao, Yandi Liu, Shiwu Zhang, Muran Li

**Affiliations:** ^1^Nankai University School of Medicine, Nankai University, 300071 Tianjin, China; ^2^Department of Gastroenterology, Tianjin Union Medical Center, 300121 Tianjin, China; ^3^Department of Pathology, Tianjin Union Medical Center, 300121 Tianjin, China

## Abstract

**Background:**

RNF180 is a tumor suppressor gene involved in cell development, proliferation, and apoptosis. Methylation of RNF180 (mRNF180) leads to low expression of RNF180, which is closely related to the occurrence and development of gastric cancer (GC). This study was designed to evaluate the potential performance of plasma mRNF180 as noninvasive biomarker for the diagnosis of GC.

**Methods:**

A total of 156 participants, including 60 patients with GC, 39 with chronic superficial gastritis (CSG), 27 with chronic atrophic gastritis (CAG), and 30 with gastric ulcer (GU) were recruited for this study. Plasma mRNF180 level was measured using real-time polymerase chain reaction.

**Results:**

As a diagnostic target, mRNF180 had a sensitivity of 71.67% (95% CI: 58.36%–82.18%) and specificity of 59.38% (95% CI: 48.85%–69.14%). The area under the ROC curve value of mRNF180 was 0.731 (95% CI: 0.648%–0.813%) for differentiation of GC from benign gastric diseases (BGD). The effectiveness of mRNF180 was superior to that of CEA, CA199, and CA724. mRNF180 was positively correlated with age, tumor size, T stage, N stage, M stage, and clinical stage of patients with GC.

**Conclusions:**

Plasma mRNF180 might serve as a useful and noninvasive biomarker for the diagnosis of GC and can be used to evaluate its prognosis.

## 1. Introduction

Gastric cancer (GC) is a malignant tumor with high morbidity and mortality. 2018 global cancer statistics released by IARC pointed out that GC is currently the fifth most common malignant disease and the third leading cause of cancer death [1]. High mortality rate is mainly due to the late discovery. About 80% of patients with GC are in advanced stages at first diagnosis, 5-year overall survival is only about 30-40% of advanced GC even if they receive comprehensive treatment [2], while 5-year overall survival of patients with early GC can exceed 90% [3]. Therefore, early diagnosis and treatment are the key to improve prognosis. Currently, gastroscopy combined with pathological diagnosis is the “gold standard” for GC diagnosis, but it is technically complex and compliance is poor, especially for asymptomatic individuals. Meanwhile, it has been reported that the clinical serum tumor markers, such as carcinoembryonic antigen (CEA), carbohydrate antigen 199 (CA199), and carbohydrate antigen 724 (CA724), have a sensitivity of 20.1-27.6%, and the combination sensitivity is 48.2% [4]. These methods are either complex in technology or low in sensitivity and specificity. It is urgent to explore a simple method with high sensitivity and specificity to make up for the limitations of the abovementioned methods.

Epigenetic and genetic alterations contribute to GC initiation and progression. Different from genetics, epigenetics does not involve in the change of DNA sequence and is potentially reversible and heritable [5]. DNA methylation is a kind of epigenetic alteration. In normal cells, most CpG (cytosine-phosphoric-guanylic) dinucleotides are scattered throughout the genome and are usually methylated, while some CpG dinucleotides aggregate into CpG islands and are rarely methylated. However, in tumor cells, it is characterized by hypomethylation of the whole genome and hypermethylation of localized promoter CpG island [6]. DNA methylation inhibits gene expression in two ways. DNA methylation will change gene conformation, unable to bind transcription factors, and bind methylated CpG-binding domain proteins instead. The latter in turn recruit other proteins and finally form compact and inactive abnormal chromatin, inhibiting gene expression and promoting tumorigenesis [5, 6]. DNA methylation is usually an early event of carcinogenesis and occurs more frequently than gene mutations [7, 8]. Therefore, as a cancer-specific marker, DNA methylation may be better than DNA mutation.

Ring finger protein 180 (RNF180) is an E3 ubiquitin ligase that plays a key role in the function of the ubiquitin-proteasome system by determining the specificity and timing of ubiquitination and subsequent degradation of its substrates [9, 10]. As a tumor suppressor gene, RNF180 is involved in a variety of physiological and pathological processes and plays an important role in cell signal transduction, apoptosis, gene transcription, and DNA repair by mediating protein degradation [9, 11]. When the body is affected by various physical, chemical, and biological factors, RNF180 is methylated, which could decrease its expression level or produce abnormal proteins, thereby possibly inducing the occurrence of a series of diseases, such as malignant tumors [12–16]. Here, we measured plasma mRNF180 levels in patients with GC, CSG, CAG, and GU and compared the sensitivity and specificity of mRNF180 to tumor markers. We also analyzed the correlation between mRNF180 *Δ* cycle threshold (*Δ*Ct) values and clinicopathological characteristics. This study may provide valuable information for the screening, diagnosis, and targeted therapy of GC.

## 2. Materials and Methods

### 2.1. Patient Recruitment, and Ethical Consideration

A total of 156 pretreatment plasma specimens, including those of 60 patients with GC, 39 with CSG, 27 with CAG, and 30 with GU were collected from the Tianjin Union Medical Center from August 2020 to August 2021. All participants met the following criteria: (1) complete case data; (2) definitive gastroscopy and pathological diagnosis; (3) no history of malignant tumor in other organs; (4) plasma samples were collected before surgery, chemotherapy, or radiotherapy; and (5) completed the whole process of sample collection. The patients' clinical characteristics, including sex, age, tumor location, tumor size, cTNM stage, and differentiation type, were recorded. The cTNM staging of GC was based on the 8th edition of the American Joint Committee on Cancer. This study was approved by the moral and ethics committee of Tianjin Union Medical Center, and informed consent was obtained from all participants.

### 2.2. Colonoscopy and Pathological Examinations and Detection of Serum Tumor Markers

Gastroscopy and pathological examinations were performed. All detailed findings, including neoplastic and nonneoplastic lesions and the size and location of the detected lesions, were recorded. Diagnosis was made based on biopsy samples from gastroscopy if patients were recommended for gastroscopy examination without subsequent surgery. Biopsy samples from surgery were used for pathological diagnosis of patients who underwent surgery. CEA, CA199, and CA724 were all detected using Roche E-70 electrochemiluminescence immunoassay analyzer and Roche E-70 special kit. CEA, CA199, and CA724 were defined as positive at the value of 5.0 ng/mL, 37.0 U/mL, and 6 U/mL, respectively.

### 2.3. Sample Collection, Processing, and Storage

A peripheral blood sample (10 mL) was collected using 10 mL BD Vacutainer®K2E (EDTA) anticoagulant tubes for RNF180 gene methylation assays. Blood samples were centrifuged for 12 min at 1350 ± 150 rcf, and the plasma was collected in a 15 mL centrifugal tube. The plasma was centrifuged again for 12 min at 1350 ± 150 rcf, and 3.5 mL supernatant was collected in a centrifuge tube. Blood samples were collected and processed at 2°C–8°C on the same day within 8 h. Plasma samples were stored at −15°C to −25°C before subsequent cfDNA (cell-free DNA) extraction. The RNF180 gene methylation assay was performed within 2 weeks after the samples were collected.

### 2.4. cfDNA Extraction and Bisulfite Conversion

Plasma cell-free DNA extraction and bisulfite conversion were performed using nucleic acid extraction kit (BioChain Science and Technology, Inc. Beijing, China) according to the manufacturer's instructions. Briefly, the extraction of DNA contained in patient plasma is based on the binding of cfDNA to magnetic particles; then, the unmethylated cytosine was transformed to uracil, while methylated cytosine remains unchanged. After washing and elution, bisulfite-modified DNA (BisDNA) was obtained. If BisDNA was not used for RNF180 gene methylation assay immediately, it can be stored at 2 to 8°C for 24 h or -25 to -15 for 72 h.

### 2.5. RNF180 Gene Methylation Assay

The Diagnostic Kit for RNF180 Gene Methylation is a qualitative assay for the real-time polymerase chain reaction (RT-PCR) detection of mRNF180 DNA in BisDNA from plasma samples. The assay carried out followed manufacturer's instructions. All kits were provided by BioChain (Beijing) Science and Technology, Inc. Beijing, China. Briefly, Each BisDNA sample (patient sample, or positive control, or negative control) was tested in triplicate. The PCR program was set as follows: activation at 94°C for 20 min; 45 cycles at 62°C for 5 s, 55.5°C for 35 s, and 93°C for 30 s; and cooling at 40°C for 5 s.

ACTB (*β*-actin) served as an internal control to assess the quantity of the input DNA and the validity of the sample preparation. Results were considered valid when the ACTB Ct was ≤34.8, and the external negative and positive controls met the validity criteria specified by the manufacturer. If mRNF180 ΔCt (Ct_RNF180_ − Ct_ACTB_) ≤ 9, the result was positive. If ΔCt > 9 or an undetermined Ct value, the result was negative. The 2/3 algorithm was used for data interpretation in this study.

### 2.6. Statistical Analysis

Statistical analyses were performed using SPSS version 26 software and GraphPad Prism version 8.3 software. The mRNF180 mean *Δ*Ct value of GC and BGD groups were compared by independent sample *t*-tests. The difference of positive detection rate between mRNF180 and serum tumor markers were evaluated by the McNemer test and Kappa test. Clinicopathological characteristics of the GC group were analyzed by the *χ*^2^ test or Fisher's exact test. Binomial distribution was assumed for calculations of 95% confidence interval (CI). Receiver operating characteristic (ROC) curves were plotted using the mean *Δ*Ct value of mRNF180 from GC and BGD groups. Ct values were set as 45 (the maximal PCR cycle number) for the undetermined samples as described previously. Area under the ROC curve (AUC) was calculated. *P* < 0.05 was considered statistically significant.

## 3. Results

### 3.1. Methylation Status of RNF180 in Plasma DNA within Different Groups

To determine whether the DNA methylation statue of RNF180 in plasma samples had diagnostic value for GC, the positive rate of 60 patients with GC, 39 with CSG, 27 with CAG, and 30 with GU was analyzed (Table 1 and Figures 1(a) and 1(b)). The positive detection rate of mRNF180 was significantly higher in the GC group than in the CSG (71.67% vs. 33.33%, *P*≦0.001) and CAG (71.67% vs. 29.63%, *P*≦0.001) group, but not in the GU group (71.67% vs. 60.00%, *P* = 0.264). When mRNF180 mean *Δ*Ct value of three PCR results were analyzed, significant results were also obtained between GC and CSG (8.13 ± 3.56 vs. 11.77 ± 2.93, *P*≦0.001) and CAG (8.13 ± 3.56 vs. 11.40 ± 2.21, *P*≦0.001) groups, but not between the GC and GU groups (8.13 ± 3.56 vs. 9.51 ± 2.71, *P* = 0.065).

### 3.2. Diagnostic Value of Plasma mRNF180 in Patients with GC

To evaluate the diagnostic value of mRNF180, the CSG, CAG, and GU groups were treated as one BGD group (Table 2). Plasma mRNF180 had 71.67% sensitivity, 59.38% specificity, 52.44% positive predictive value (PPV), and 77.03% negative predictive value (NPV). Despite the unsatisfactory specificity, the sensitivity of more than 70% is still higher than that of most serum biomarkers. Thus, plasma mRNF180 can be used as a screening test, especially for those with poor basic conditions who are unable to tolerate gastroscopy.

To achieve the observed test performance, ROC curve analysis was performed to evaluate the AUC, sensitivity, and specificity and to determine the best cut-off value of mRNF180 for GC diagnosis. As shown in Table 3 and Figure 2, mRNF180 had an AUC of 0.731 (95% CI 0.648–0.813), and sensitivity and specificity were 79.96% and 65.00%, respectively, at the *Δ*Ct cut-off value of 9.21. Those results showed that plasma mRNF180 demonstrated a remarkable performance in the diagnosis of GC. In addition, when mRNF180 *Δ*Ct value is lower than 9.21, doctors should suggest gastroscopy to rule out malignant lesions. In this study, mRNF180 *Δ*Ct value of ≤9 was considered positive, which was close to the cut-off value calculated using the Youden index.

### 3.3. Comparison of the Predictive Power of mRNF180, CEA, CA199, and CA724 for GC Detection

CEA was found in 17 of 60 patients with GC and 4 of 96 control patients. In addition, CA199 was found in 16 of 60 patients with GC and 7 of 96 control patients. Similarly, CA724 was found in 17 of patients with 60 GC and 11 of 96 control patients. Thus, the sensitivities of CEA, CA199, and CA724 were 28.33%, 26.67%, and 28.33%, respectively, which were all lower than that of mRNF180 (Table 2). Regarding AUC for GC, the area of mRNF180 was larger than that of CEA, CA199, and CA724 (Table 3 and Figure 2).

To compare the predictive power between mRNF180 and serum tumor markers during the auxiliary diagnosis of GC, additional McNemer test and Kappa test were conducted in the GC group, and the results showed that the overall agreement was poor between both tests (Kappa values ranged from -0.010 to 0.196), and the positive rate of mRNF180 was significantly higher than that of CEA (*P*≦0.001), CA199 (*P*≦0.001), and CA724 (*P*≦0.001). (Table 4 and Figure 3). These data indicate that mRNF180 assay was specific for GC detection and better than CEA, CA199, and CA724.

### 3.4. Correlation of Pretreatment Plasma mRNF180 with the Clinicopathological Characteristics of GC

Data on the clinicopathological characteristics of the GC group were collected to study the specific correlation between peripheral mRNF180 and pathological manifestations. Detailed clinicopathological characteristics are summarized in Table 5 and Figures 4(a) and 4(b). We observed that the mRNF180-positive rate was significantly upregulated in advanced T stage (Tis/1/2/3 vs. T4, *P* = 0.005) and N stage (N0/1 vs. N2/3, *P* = 0.001). There were no significant differences among mRNF180-positive rate and age, sex, tumor location, tumor size, differentiation, M stage, or clinical stage. We further explored the relationship between mean mRNF180 *Δ*Ct values and clinicopathological characteristics. In contrast to the analysis of mRNF180 positivity, mRNF180 mean *Δ*Ct value was positively correlated with age (*P* = 0.010), tumor size (*P* = 0.033), T stage (*P* = 0.004), N stage (*P*≦0.001), M stage (*P* = 0.011), and clinical stage (*P* = 0.022), but not with sex, tumor location, or differentiation (*P* > 0.05). These results suggest that mRNF180 is involved in the formation of the malignant biological behavior of GC and may be used to predict its aggravation.

## 4. Discussion

Previous studies have focused on the expression of RNF180 mRNA and protein in GC tissues. Cheung et al. found that the RNF180 protein was significantly downregulated in GC tissues compared with in adjacent nontumor tissues [17]. Han et al. collected tissue samples for research and found that average methylation rates, methylated CpG site counts, and hypermethylated CpG site counts of RNF180 increased gradually with disease severity (GC>CAG>CON) [18], suggesting that the production of mRNF180 is an early event in gastric carcinogenesis and may be involved in the initiation of cellular transformation from normal cells into tumors. In addition, the authors of this and other studies have proposed that the expression of RNF180 in GC tissues is negatively related to the number of metastatic lymph nodes and overall survival [19, 20]. Further, experiments on animals and cell lines suggest that RNF180 inhibits the proliferation, migration, and invasion of GC cells and inhibits tumor growth and lymphangiogenesis [20, 21]. Considering the accessibility of sample acquisition, detecting DNA methylation in peripheral blood undoubtedly provides a new method for noninvasive detection of GC.

In Cheung's study, plasma mRNF180 was detected in 56% (18/32) of patients with GC, but not in 64 healthy controls (AUC of 0.685) [17]; in Zhang's study, mRNF180 was detected in 57.89% (33/57) of patients with GC and in 23.81% (10/42) of the controls [22]. In Cao's study, mRNF180 was detected in 32.4% (24/74) of patients with EGC, 13.1% (13/99) of BGD patients, and 5.3% (3/57) of healthy controls (AUC of 0.636) [23]. However, in our study, mRNF180 was detected in 71.67% (43/60) of patients with GC and in 40.63% (39/96) of the controls with 71.67% sensitivity and 59.38% specificity. Although the sensitivity was higher than that previously reported, the specificity was relatively lower. This was because our study was conducted under the background of opportunistic screening, which was different from screening an average-risk population; the probability of GC detection by opportunistic screening is higher [24], i.e., the false positive rate of BGD is higher than that of healthy controls. Besides, the mRNF180-positive rate in GU was 60.00% compared to 71.67% in GC, which was much higher than the positive rate in CSG and CAG. This contributes to the low specificity and makes mRNF180 marker not GC specific. Compared with CSG and CAG, the blood supply of GU and GC is relatively higher. And cfDNA from healthy individuals is comprised mostly of DNA released by dead hematopoietic cells [25]. Therefore, mRNF180 is more likely to be released into the bloodstream. Future studies will investigate whether the mRNF180 positive rate is associated with blood supply.

Furthermore, Zhang et al.'s study highlighted that mRNF180 was positively correlated with tumor size, differentiation, clinical stage, N stage, and M stage [22]. Cao et al. found no correlation between mRNF180 and clinicopathological characteristics [23]. However, our study suggests that the mRNF180-positive rate was significantly associated with T stage and N stage (*P* < 0.05), but no significant difference in positivity was found among age, sex, tumor location, tumor size, differentiation, M stage, or clinical stage in GC (*P* > 0.05), although there was a trend of positivity for stage 0/I/II being lower than that of later stages (*P* = 0.051). The mRNF180 mean *Δ*Ct value was significantly associated with age, tumor size, T stage, N stage, M stage, and clinical stage (*P* < 0.05), but not with sex, tumor location, or differentiation (*P* > 0.05). Notably, the *P* value of differentiation is 0.057, which is close to 0.05. If the sample size is further expanded, different results may be obtained. Compared with previous studies, the main difference in our study is that mRNF180 is age related in GC. Similarly, age-related mRNF180 detection difference was also observed in GU, CSG, and CAG. Studies have described this possibility, and age-related detection can be found in many methylation markers [26, 27].

Notably, Cao et al. assessed mSEPT9 and mRNF180 for noninvasive diagnosis of EGC and found that the positive rate of combined mSEPT9 and mRNF180 was the highest, followed by mRNF180, mSEPT9, CA724, CA125, CEA, and CA199 [23], which was consistent with our study. The positive rate of mRNF180 was superior to that of CEA, CA199, and CA724. The mRNF180 definitely complemented the diagnosis of serum tumor marker-negative GC patients with a remarkable discrimination performance. However, in Cao et al.'s study, there was no correlation between mRNF180 and Lauren classification, histologic grade, N stage, and depth of invasion, which was different from the present findings. The different results may have resulted from the experimental group of the latter study being early stage, with the invasive behavior not showing yet in most of the patients. As the disease advances, tumor cells gradually infiltrate deep tissues, blood vessels, and lymph nodes, and more mRNF180 will be released into circulation.

These data clearly show that the mRNF180 assay alone can detect GC with high sensitivity. However, we must acknowledge that the specificity was not satisfactory. In Zhang et al.'s study, when mRNF180 was combined with mSFRP2, the sensitivity of the combined test improved, but the specificity did not improve [22]. However, in Cao et al.'s study [23], in which mRNF180 was combined with mSEPT9, the sensitivity of the combined test improved, and the specificity remained satisfactory. One strategy for improving GC diagnosis is to combine multiple methylation biomarkers. In colorectal cancer, mSEPT9 can be used as a tumor biomarker to diagnose the disease and predict the risk of prognosis, recurrence, and metastasis, and its value has been confirmed in clinical practice [28, 29]. Since colorectal cancer and GC are both gastrointestinal tumors, they share some common molecular characteristics [30], and the value of mSEPT9 detection for screening GC will attract attention. Besides, global methylation profiling has been reported to identify cancer-specific methylation signatures [25, 31]. GC-specific DNA methylation also could be identified by the analysis of whole-genome scale DNA methylation data. Further studies are warranted to identify more biomarkers and refine the best panel for GC detection. Improving the detection accuracy by optimizing the methylation detection technology and exploring the specific signal pathway mechanisms underlying methylation oncogenic effects will be the focus of future investigations.

There are some limitations to the present study. First, although our results showed that mRNF180 was associated with T stage, N stage, M stage, and clinical stage, the number of patients was limited, and bias might have occurred. Second, the controls we used may not be appropriate. Third, we did not validate the status of mRNF180 in GC tissues. In the future, we will enroll more patients, including healthy controls, and further studies in tissue and plasma samples would be performed to validate these findings. Also, we will further explore the causes of the high positive rate of GU.

In summary, mRNF180 had a sensitivity of 71.67% and specificity of 59.38%. Although the specificity was relatively lower, the sensitivity of 71.67% was encouraging. More studies are needed to improve the specificity to make mRNF180 be considered useful and noninvasive biomarkers for diagnosing GC and distinguishing between benign and malignant diseases of the stomach, especially for patients with poor basic conditions who are unable to tolerate gastroscopy. In addition, mRNF180 were associated with T stage, N stage, M stage, and clinical stage, and this can be used to evaluate the malignancy and prognosis of GC.

## Figures and Tables

**Figure 1:** Positive rate and mean *Δ*Ct value of mRNF180 in each enrolled group. (a) Positive detection rate of mRNF180 for each enrolled group. Positive detection rate was compared by the *χ*^2^ test or Fisher exact test. (b) The mRNF180 mean *Δ*Ct value for each enrolled group. Mean *Δ*Ct value was compared by *t*-test. The mRNF180 *Δ*Ct cut-off value = 9.21 was calculated by the Youden index. GC: gastric cancer; CSG: chronic superficial gastritis; CAG: chronic atrophic gastritis; GU: gastric ulcer.

**Figure 2:** ROC curve of mRNF180 and serum tumor markers. The mRNF180 had an AUC of 0.731, CEA had an AUC of 0.583, CA199 had an AUC of 0.606, and CA724 had an AUC of 0.621. AUC (RNF180) > AUC (CA724) > AUC (CA199) > AUC (CEA).

**Figure 3:** Positive rates of mRNF180 and serum tumor markers in the GC group. Positive detection rate was compared by McNemer test. ns: not significant.

**Figure 4:** Correlations between mRNF180 and clinicopathological characteristics of the GC group. Clinicopathological characteristics include sex, age, tumor location, tumor size, T stage, M stage, N stage, clinical stage, and differentiation. (a) Positive detection rate was compared by the *χ*^2^ test or Fisher exact test. (b) Mean *Δ*Ct value was compared by *t*-test or *F* test. ns: not significant.

**Table 1:** Mean *Δ*Ct value and positive rate of mRNF180 in each enrolled group.

Groups	*N*	Positive		Mean *Δ*Ct value	
		Number	%	Mean	Std. deviation
GC	60	43	71.67	8.13	3.56
CSG	39	13	33.33	11.77	2.93
CAG	27	8	29.63	11.40	2.21
GU	30	18	60.00	9.51	2.71
*P* ^∗^		≦0.001		≦0.001	
*P* ^∗∗^		≦0.001		≦0.001	
*P* ^∗∗∗^		0.264		0.065	

*P* ^∗^ compared with CSG, *P*^∗∗^ compared with CAG, and *P*^∗∗∗^ compared with GU. GC: gastric cancer; CSG: chronic superficial gastritis; CAG: chronic atrophic gastritis; GU: gastric ulcer.

**Table 2:** Sensitivity, specificity, PPV, and NPV of mRNF180 and serum tumor markers.

	Sensitivity (95% CI)	Specificity (95% CI)	PPV (95% CI)	NPV (95% CI)
mRNF180	71.67 (58.36-82.18)	59.38 (48.85-69.14)	52.44 (41.18-63.47)	77.03 (65.52-85.68)
CEA	28.33 (17.82-41.64)	95.83 (89.07-98.66)	80.95 (57.42-93.71)	68.15 (59.50-75.75)
CA199	26.67 (16.45-39.89)	92.71 (85.06-96.77)	69.57 (46.99-85.94)	66.92 (58.16-74.68)
CA724	28.33 (17.82-41.64)	88.54 (80.02-93.86)	60.71 (40.73-77.87)	66.41 (57.45-74.36)

PPV: positive predictive value; NPV: negative predictive value.

**Table 3:** Area under ROC (AUC).

Groups	AUC (95% CI)	Std. error	Asymptotic sig.	Cut-off value	Sensitivity (95% CI)	Specificity (95% CI)
mRNF180	0.731 (0.648-0.813)	0.042	<0.0001	9.21	73.96 (64.38-81.69)	65.00 (52.36-75.83)
CEA	0.583 (0.484-0.681)	0.050	0.0826	4.54	31.67 (21.31-44.23)	94.79 (88.38-97.76)
CA199	0.606 (0.513-0.699)	0.048	0.0260	45.20	25.00 (15.78-37.23)	95.83 (89.77-98.37)
CA724	0.621 (0.523-0.714)	0.048	0.0115	2.10	60.00 (47.37-71.43)	66.67 (56.76-75.29)

**Table 4:** Comparison of positive rates of mRNF180 and serum tumor markers in the GC group.

	Positive rate	*P*	Kappa value
mRNF180	71.67% (43/60)	—	—
CEA	28.33% (17/60)	≦0.001	-0.010
CA199	26.67% (16/60)	≦0.001	0.196
CA724	28.33% (17/60)	≦0.001	0.046

**Table 5:** Correlations between mRNF180 and clinicopathological characteristics of the GC group.

Clinicopathological characteristics	mRNF180					
	*N*	Positive	Negative	*P*	Mean *Δ*Ct value	*P*
Sex				1.000		0.746
Male	44	31	13		8.22	
Female	16	12	4		7.88	
Age (years)				0.171		0.010
<70	34	22	12		9.15	
≥70	26	21	5		6.80	
Tumor location						
Upper third	16	11	5		NA	
Middle third	20	14	6		NA	
Lower third	18	12	6		NA	
>2/3 stomach	4	4	0		NA	
NA	2					
Tumor size (cm)				0.142		0.033
<6.0	25	16	9		9.09	
≥6.0	32	26	6		7.08	
NA	3	1	2			
T stage				0.005		0.004
Tis+T1+T2+T3	20	10	10		9.78	
T4	34	29	5		6.94	
NA	6	4	2			
N stage				0.001		≦0.001
N0+N1	23	11	12		10.28	
N2+N3	30	27	3		6.27	
NA	7	5	2			
M stage				0.463		0.011
M0	38	26	12		9.01	
M1	22	17	5		6.61	
NA	0					
Clinical stage				0.051		0.022
0+I+II	11	5	6		10.15	
III+IV	45	36	9		7.44	
NA	4	2	2			
Differentiation				0.284		0.057
High+moderate	12	6	6		10.18	
Low	32	23	9		7.73	
NA	16	14	2			

## Data Availability

The data used during the present study are available from the corresponding author upon reasonable request.
